This article has been retracted.

# Intolerance of Uncertainty Scale-12: Psychometric Properties of This Construct Among Iranian Undergraduate Students

**DOI:** 10.3389/fpsyg.2022.894316

**Published:** 2022-06-08

**Authors:** Balachandran Vadivel, Zahra Azadfar, Mansor Abu Talib, Dhameer A. Mutlak, Wanich Suksatan, Abbas Abd Ali Abbood, Mohammed Q. Sultan, Kelly A. Allen, Indrajit Patra, Ali Thaeer Hammid, Abbas Abdollahi, Supat Chupradit

**Affiliations:** ^1^Department of English, Cihan University - Duhok, Duhok, Iraq; ^2^Department of Psychology, Faculty of Educational Sciences and Psychology, Alzahra University, Tehran, Iran; ^3^Department of Psychology, Faculty of Social Sciences and Liberal Arts, UCSI University, Kuala Lumpur, Malaysia; ^4^Al-Nisour University College, Baghdad, Iraq; ^5^Faculty of Nursing, HRH Princess Chulabhorn College of Medical Science, Chulabhorn Royal Academy, Bangkok, Thailand; ^6^Department of Business Administration, Al-Mustaqbal University College, Hillah, Iraq; ^7^College of Dentistry, Al-Ayen University, Nasiriyah, Iraq; ^8^Educational Psychology and Inclusive Education, Faculty of Education, Monash University, Clayton, VIC, Australia; ^9^Independent Researcher, Durgapur, India; ^10^Computer Engineering Department, Imam Ja’afar Al-Sadiq University, Baghdad, Iraq; ^11^Department of Counseling, Faculty of Education and Psychology, Alzahra University, Tehran, Iran; ^12^Department of Occupational Therapy, Faculty of Associated Medical Sciences, Chiang Mai University, Chiang Mai, Thailand

**Keywords:** IUS-12, intolerance of uncertainty scale-12, Iranian, psychometrics, reliability, undergraduate students

## Abstract

**Background:**

Uncertainty intolerance (IU), the tendency to think or react negatively toward uncertain events may have implication on individuals’ mental health and psychological wellbeing. The Intolerance of Uncertainty Scale-12 (IU-12) is commonly used across the globe to measure IU, however, its’ psychometric properties are yet to be evaluated in Iran with a Persian-speaking population. Therefore, the purpose of this research was to translate and validate the IU-12 among Iranian undergraduate students.

**Materials and Methods:**

The multi-stage cluster random sampling was employed to recruit 410 Iranian undergraduate students (260 females) from the Azad University to complete the IU-12, the Depression Anxiety Stress Scale-2, and the Penn State Worry Questionnaire in a cross-sectional design. In this study, face validity, content validity, construct validity, and concurrent validity were measured and Construct Reliability (CR) and Cronbach’s alpha were used to measure reliability.

**Results:**

The impact score of the translated IU-12 indicated acceptable face validity (value of impact score was greater than 1.5). The value of Content Validity Index (CVI) and the value of Content Validity Ratio (CVR) were above 0.7 and 0.78, respectively. The values of CVI and CVR indicated the items had acceptable content validity and were deemed essential to the measure. The measurement model analysis showed the measure with two subscales had good fit indices (CMIN/*df* = 2.75, *p* < 0.01, RMSEA = 0.07, TLI = 0.94, CFI = 0.95, GFI = 0.94). A Confirmatory Factor Analysis (CFA) indicated the scale was composed of the two subscales found in the English-version of the scale (prospective anxiety and inhibitory anxiety), and no items were removed from the scale. The values of CR (0.86) and Cronbach’s alphas (0.89) showed the measure had appropriate internal consistency.

**Conclusion:**

The findings support the psychometric properties of the Persian version of the IU-12. This scale could be used to reliably and accurately measure uncertainty intolerance among undergraduate students in Iran.

## Introduction

The academic environment of a university can be challenging and demanding for students. Undergraduate students often experience high levels of stress or uncertainty over academic tasks, maintaining interpersonal relationships, or planning their career trajectory (Nekić and Mamić, 2019). In addition, the onset of a number of psychological disorders occur in early adulthood when individuals are experiencing university for the first time (Kessler et al., 1998). Epidemiology studies report that nearly half of undergraduate students meet DSM-V criteria for at least one mental illness (American Psychiatric Association, 2013). The prevalence rates of anxiety and depression symptoms are estimated to be 20 and 7% in university students, respectively (Blanco et al., 2008). Test anxiety also is common in undergraduate students and individuals with high levels of test anxiety are more likely to engage in IU and worry and may see failing as intolerable and threatening (Huntley et al., 2020). Given the degree of potential instability and uncertainty in academic settings, IU is a risk factor in the development of mental health problems among undergraduate students (Nekić and Mamić, 2019). Therefore, a valid and reliable measure for assessing IU among undergraduate students is necessary in order to assist prevention and intervention programs.

Uncertainty intolerance is defined as a dispositional tendency to react negatively to unpredictable events and ambiguous and unknown situations (Carleton et al., 2007; Birrell et al., 2011; Wilson et al., 2020). According to past research, greater IU is associated with poor decision-making, diminished coping skills, low motivation, avoidance of ambiguous situations, and a reduction in academic performance (Dugas, 1997; Jacoby et al., 2015). Although, IU is also well-known to be a central factor in the intolerance of uncertainty model (IUM) that explains General Anxiety Disorder (GAD) (Dugas et al., 1998), several studies have supported its role as a transdiagnostic factor in a range of psychological disorders, such as depression, anxiety, and stress (Boelen and Lenferink, 2018; Rosser, 2019; Swee et al., 2019). Accordingly, Carleton (2016) defined IU as the incapacity to endure the perception of uncertainty. Hong and Cheung (2015) indicated that IU is correlated with various cognitive vulnerabilities including susceptibility to anxiety, fear of negative appraisal, and ruminative-thinking styles. Hence, IU may account for high comorbidity across different disorders, such as anxiety, stress, and depression (Boswell et al., 2013; Abdollahi et al., 2019). Previous studies on the relationship between IU and psychopathology demonstrated that IU is negatively related to symptoms of post-traumatic stress disorder (Oglesby et al., 2015), social anxiety disorder (Whiting et al., 2014), panic disorder and agoraphobia (Carleton et al., 2013), obsessive-compulsive disorder (Jacoby et al., 2013), health anxiety (Wright et al., 2016), and eating pathologies (Kesby et al., 2017).

To date, the Intolerance of Uncertainty Scale (IU-12) has demonstrated excellent psychometric properties for assessing IU as a transdiagnostic risk factor in clinical and non-clinical populations (Carleton et al., 2007). The IU with 12-item is a short form of the IU with 27-items (Freeston et al., 1994) and the most common self-report measure for assessing negative perceptions and reactions to equivocal situations, uncertainty, and future events (Carleton et al., 2007). Freeston et al. (1994) initially introduced the IU-27 as a five-factor measure that investigated: unacceptability and avoidance of uncertainty, negative social evaluation caused by uncertainty, uncertainty-related frustration, uncertainty causing stress, and uncertainty preventing action. The IU-12 was developed to remove some GAD-specific items. The IU-12 has a stable two-factor structure that is comprised of two sub-scales, indicating both anxious and avoidant components of IU. Prospective IU (the cognitive component) refers to the tendency to cognitive predict future events and actively search out information to help reduce uncertainty. Inhibitory IU (the behavioral component) refers to behavioral inhibition or avoidance in the face of uncertainty (Carleton et al., 2007). An Australian study compared the IU-12 to the IU-27, and the results showed that there was no difference between the IU-12 and the IU-27 in terms of internal consistency and test-retest reliability (Khawaja and Yu, 2010). The shortness of the IU-12 made it more applicable in different settings and the removal of the GAD-specific items improved its use in measuring IU amongst a more diverse group of individuals.

The English version of the IU-12 (Carleton et al., 2007) has been validated with two samples. The first sample consisted of 254 undergraduate students aged 19–37 and 193 women aged 18–50 years old. The second group included 818 undergraduate students. Findings supported a two-factor structure (prospective anxiety and inhibitory anxiety), acceptable internal consistency, and high correlation with the original IU [*r* = 0.96; (Carleton et al., 2007)]. This scale has also been validated in clinical and non-clinical populations including children in the United Kingdom (IU-C) (Osmanağaoğlu et al., 2021), outpatients with psychosis in Pennsylvania (Bredemeier et al., 2019), undergraduate students in the United Kingdom (Huntley et al., 2020), and individuals with GAD in Australia (Wilson et al., 2020). The aforementioned studies have demonstrated good internal consistency values for IU-12 with Cronbach’s alpha values between 0.82 and 0.96 (Carleton et al., 2007; Bredemeier et al., 2019; Huntley et al., 2020; Wilson et al., 2020; Osmanağaoğlu et al., 2021). In addition, the IU-12 positively correlated with depression, anxiety, state worry, and GAD, indicating acceptable convergent validity (Carleton et al., 2007). Other psychometric studies using factor analysis method achieved two subscales same as the original study (Huntley et al., 2020; Wilson et al., 2020).

Validation of a measure with sufficient psychometric properties can help screen undergraduate students for emotional problems in order to design prevention programs and clinical interventions. Additionally, the shorter IU has the potential to encourage a broader evaluation of IU. As all of the psychometric studies of the IU-12 have been conducted in western countries, there is a need to evaluate the validity and reliability of the IU-12 in other countries, including Iran. Currently, only the IU-27 is used in Iran to measure IU in adults (Freeston et al., 1994). As such, the current study aims to measure the psychometric properties of the Persian version of IU-12 among Iranian university students. In addition, this study considers the results of previous studies on the Penn State Worry Questionnaire (PSWQ) (Meyer et al., 1990) and the Depression Anxiety Stress Scales (DASS-21) (Antony et al., 1998) in order to measure the concurrent validity of the Persian version of the IU-12 scale. We hypothesize that the scores of the Penn State Worry Questionnaire (PSWQ) (Meyer et al., 1990) and the Depression Anxiety Stress Scales (DASS-21) (Antony et al., 1998) would positively correlate with the IU-12 scores among university students.

## Materials and Methods

### Participants

Participants were 410 university students, of which 260 were females and 150 were males. The participants ranged in age from 18 to 24 years old (*M* = 22.12, *SD* = 2.15). Of the total participants, 350 (85%) were single and 60 (15%) were married. There were 127 (31%) participants from medical fields, 115 (28%) participants were from technical fields, and 168 (41%) participants were from social science fields. In terms of academic year, 131 (32%) students were in the first year of university, 143 (35%) students were in the second year of university, 74 (18%) students were in the third year of university, and 62 (15%) students were in the last year of university.

### Instruments

#### The Intolerance of Uncertainty Scale-12 (Carleton et al., 2007)

This measure consists of 12 items (e.g*., “It frustrates me not having all the information I need”*) and utilizes a 5-point Likert scale from 1 (“*Not at all characteristic of me*”) to 5 (“*Very Characteristic of me*”) to evaluate two sub-scales of IU (prospective anxiety and inhibitory anxiety). A greater score in each subscale indicates a greater level of prospective anxiety and inhibitory anxiety. A previous study reported an acceptable internal consistency with a Cronbach’s Alpha of 0.93 (Wilson et al., 2020).

To translate the English version of the IU-12 measure into Persian, the Brislin (1986) translation method was employed. Two experienced translators who were fluent in English and Persian were independently invited. One translator first conducted the translation of the IU-12 measure from English into Persian. The second translator was then asked to back-translate the resulting Persian IU-12 measure from Persian into English, unaware of the first translation operation. Finally, three independent translators compared the two versions and no major variations in terms of content and concept between the Persian version and the original measure were found.

#### Depression Anxiety Stress Scale-21 (Lovibond and Lovibond, 1996)

This measure consists of 21 items (e.g., *“depression: I found it difficult to work up the initiative to do things,” “anxiety: I felt scared without any good reason,” and “stress: I found it hard to wind down”*) that uses a 4-point Likert scale from 0 *(“Did not apply to me at all”)* to 3 *(“Applied to me very much, or most of the time”*) to evaluate depression, anxiety, and stress. A greater score in each subscale indicates a greater level of depression, anxiety, and stress. An Iranian version of this measure was validated in 2008 and used in this study. The results showed the DAS-21 had acceptable internal consistency with Cronbach’s Alphas ranging from 0.79 to 0.90 (Asghari et al., 2008). In this study, the Cronbach’s Alphas for depression, anxiety and stress were 0.81, 0.86, and 0.89, respectively.

#### The Penn State Worry Questionnaire (Meyer et al., 1990)

This measure consists of 16 items (e.g*., “Many situations make me worry.”*) and uses on a 5-point Likert scale from 1 (*“not at all typical of me”*) to 5 (“*typical of me*”) to evaluate engagement of worry and absence of worry. Items 1, 3, 8, 10, and 11 must be reverse coded and a greater score in this scale indicates a greater level of worry. An Iranian version of this measure was validated in 2010 and used in this study. The results showed the PSWQ had an acceptable internal consistency with a Cronbach’s Alpha of 0.88 (Dehshiri et al., 2010). In this study, the Cronbach’s Alphas for the PSWQ was 0.89.

### Procedure

The ethics committee of Alzahra University accepted the present study’s procedure and research materials. After reviewing the research objectives and questionnaires, Azad University permitted the distribution of the questionnaires among undergraduate students. The multi-stage cluster random sampling was employed to recruit undergraduate students in a cross-sectional design. At the first stage, thirteen faculties were divided into three clusters of social science, technical, and medicine. At the second stage, from each cluster, a faculty was randomly selected and then a class was selected based on the academic year. The questionnaires were then distributed among the students of that class after coordinating with the lecturer of the class. Written consent forms were read and signed by participants prior to completing the survey. The approximate time to complete the questionnaires was about 45 min, after which the lecturer delivered the questionnaires to the researchers. The data collection occurred from September to November 2019. Inclusion criteria for participation in this study included being a bachelor’s student, being in the age range of 18–24 years, and being willing to participate in the study.

### Data Analyses

The IU-12 was first evaluated for face validity, which is the degree to which end users agree that the items of an assessment instrument accurately reflect the targeted construct, as well as evaluating an item in terms of difficulty, ambiguity, and relevancy. Secondly, the content validity of the item was assessed by experts to what extent the items of instruments reflected intolerance of uncertainty. Thirdly, the construct validity for the IU-12 was evaluated. Confirmatory Factor Analysis (CFA) using AMOS-24 software was used to assess factor loadings, measurement fit indices, convergent validity between items and internal consistency for instrument. The Cronbach’s alpha was also measured using SPSS-26 software to assess internal consistency.

## Results

### Face Validity

An impact score index was used to estimate the face validity of the translated IU-12. Eight undergraduate students were asked to state their opinions about the relevancy, comprehension, and appropriateness of items by selecting one of the values of 5-point Likert scale, from 1 (*not important*) to 5 (*completely important*). The formula for calculating the impact score index is to multiply the frequency of participants who chose the values of 4 and 5 on the scale by the mean score of each item. If the value of the impact score is equal to or greater than 1.5 (Hajizadeh and Asghari, 2011), that impact score index provides evidence of an acceptable face validity for the item. The results of calculating the impact score index indicated that all items had values greater than 1.5, showing satisfactory face validity of the items.

### Content Validity

The Content Validity Index (CVI) and the Content Validity Ratio (CVR) were used to measure the scale’s content validity. The CVI estimates the simplicity, clarity, and relevancy of items from the experts’ point of view. Nine psychologists (i.e., experts) were asked to state their opinions about the items on a 4-point Likert scale from (1) *not relevant at all* to (4) *highly relevant*. The value of the CVI is calculated by dividing the number of experts who selected the values of 3 and 4 by the total number of experts. If the value of the CVI is equal to or greater than 0.7 the item has acceptable content validity (Cook and Beckman, 2006). The CVR estimates the essentiality of items, which the psychologists evaluated on a 3-point scale from (1) *not essential* to (3) *essential*. The value of CVR is calculated by subtracting half the number of experts (N/2) from the number of experts who selected a value of 3, then dividing this by N/2. A CVR greater than the Lawshe’s value (0.78) indicates the item has satisfactory content validity (Lawshe, 1975). As shown in Table 1, the results of CVI and CVR indicate acceptable content validity for all items.

**TABLE 1:** Content Validity Ratio and Content Validity Index for the items of intolerance of uncertainty scale-12.

No.	Items	CVI			CVR
		
		Simplicity (1–4)	Relevancy (1–4)	Clarity (1–4)	Essential (1–3)
1	Unforeseen events upset me greatly.	0.78	0.78	1	0.78
2	It frustrates me not having all the information I need.	1	1	1	1
3	One should always look ahead so as to avoid surprises.	1	1	1	1
4	A small, unforeseen event can spoil everything, even with the best of planning.	1	1	1	1
5	I always want to know what the future has in store for me.	1	1	1	1
6	I can’t stand being taken by surprise.	1	1	1	1
7	I should be able to organize everything in advance.	1	1	1	1
8	Uncertainty keeps me from living a full life.	1	1	1	1
9	When it’s time to act, uncertainty paralyzes me.	1	1	1	0.78
10	When I am uncertain, I can’t function very well.	1	1	1	1
11	The smallest doubt can stop me from acting.	1	1	1	0.1
12	I must get away from all uncertain situations.	0.78	1	1	1

### Preliminary Analysis

Preliminary data analyses were conducted using Statistical Package for the Social Science (SPSS version 24) in order to address missing data. In total, 2% of the data was missing, and all missing data were addressed using the regression imputation method. Outliers were checked by Mardia’s multivariate kurtosis test and Mahalanobis distance using AMOS 24 (Bentler and Wu, 2005). The critical ratio for Mardia’s kurtosis was 21.97 and the maximum Mahalanobis distance value was 38.72, indicating the data were normal and did not have outliers (Tabachnick and Fidell, 2012).

### Construct Validity

To estimate the construct validity, a confirmatory factor analysis in AMOS software was used to examine the hypothesized relations between the items and the factors. Hair et al. (1998) recommended a 20:1 case-to-item ratio for confirmatory factor analysis (CFA). There were 410 participants and 12 items (intolerance of uncertainty scale) in this study, and the minimal case-to-item ratio was reached. The construct validity consists of three parts:

a) Assessment of factor loading values: If the factor loading value is less than 0.4, greater than 1 or negative, it is necessary to delete the item (Tabri and Elliott, 2012). As seen in Figure 1, the values of the factor loadings did not violate these cutoffs, therefore all items were kept in the scale. At this stage, the means and standard deviations of the items were also calculated (see Table 2).
b) Assessment of the measurement model fit indices: CMIN/*df* < 5; Root Mean Squared Error of Approximation (RMSEA) < 0.08; Tucker- Lewis Index (TLI), Comparative Fit Index (CFI), and the Goodness of Fit Index (GFI) > 0.90 (Byrne, 2013). The results revealed Model B with two subscales had slightly worse fit indices (CMIN/*df* = 2.75, *p* < 0.01, RMSEA = 0.07, TLI = 0.94, CFI = 0.95, GFI = 0.94) compared to bifactor model (Model A) (CMIN/*df* = 2.61, *p* < 0.01, RMSEA = 0.07, TLI = 0.95, CFI = 0.95, GFI = 0.95). Therefore, the total score could be calculated for the IU-12 scale.
c) Assessment of convergent validity and internal consistency between items of the measure: The Average Variance Extracted (AVE) values were greater than 0.5, demonstrating appropriate convergent validity for the measure (see Table 3). Construct Reliability (CR) values and Cronbach’s alphas were also above 0.7 (see Table 3), showing the measure’s appropriate internal consistency (Byrne, 2013).

**FIGURE 1:** The intolerance of uncertainty scale-12 construct Model **(A)** (bifactor model) and the IU-12 construct Model **(B)** with two sub scales.

**TABLE 2:** Means and standard deviations of the items of intolerance of uncertainty scale-12.

No.	Items	Mean	Std. deviation
1	Unforeseen events upset me greatly.	2.76	0.94
2	It frustrates me not having all the information I need.	3.88	0.91
3	One should always look ahead so as to avoid surprises.	2.29	0.83
4	A small, unforeseen event can spoil everything, even with the best of planning.	3.56	1.1
5	I always want to know what the future has in store for me.	3.49	0.92
6	I can’t stand being taken by surprise.	3.22	0.97
7	I should be able to organize everything in advance.	3.75	1
8	Uncertainty keeps me from living a full life.	3.96	1.2
9	When it’s time to act, uncertainty paralyzes me.	3.89	0.98
10	When I am uncertain, I can’t function very well.	3.71	0.96
11	The smallest doubt can stop me from acting.	3.39	1
12	I must get away from all uncertain situations.	3.54	1.04

**TABLE 3:** Average Variance Extracted and Construct Reliability for two subscales of uncertainty intolerance.

Variable	AVE	CR	Cronbach’s alpha
Prospective anxiety	0.53	0.83	0.86
Inhibitory anxiety	0.5	0.91	0.93
Intolerance of uncertainty scale	0.51	0.86	0.89

### Concurrent Validity

The correlation analysis results indicated that two subscales of the translated IU-12 had positive relationships with worry *(r = 0.75, p < 0.001)*, stress *(r = 0.61, p < 0.001)*, anxiety *(r = 0.61, p < 0.001)*, and depression *(r = 0.54, p < 0.001)* (see Table 4).

**TABLE 4:** Correlations between the studied variables.

Variables	1	2	3	4	5	6	7
(1) Inhibitory anxiety	1						
(2) Prospective anxiety	0.89**	1					
(3) Worry	0.77**	0.73**	1				
(4) Depression	0.64**	0.67**	0.62**	1			
(5) Anxiety	0.69**	0.69**	0.68**	0.42**	1		
(6) Stress	0.63**	0.71**	0.69**	0.49**	0.73**	1	
(7) Intolerance of uncertainty scale	0.87**	0.81**	0.75**	0.54**	0.61**	0.61**	1

**, significant at the 0.01 level.

## Discussion

The aim of this study was to translate the IU-12 into the Persian language and investigate the scale’s psychometric properties using a sample of Iranian university students. The Brislin method was used to translate the IU-12 from English into the Persian language, and the translators confirmed the consistency of this Persian version with the original version. Appropriate face validity was verified by the results of the impact score index. The results of the content validity test showed that the translated items of IU-12 had the quality of simplicity, clarity, relevancy, and essentiality. Therefore, the items properly evaluated IU among Iranian university students. The results of the confirmatory factor analysis in accordance with the two factors (prospective anxiety and inhibitory anxiety) of the IU-12 scale indicated that the translated version of this measure agreed with the two factors found in the original English version, and fit the data accurately (Khawaja and Yu, 2010; Fergus and Wu, 2013; Jacoby et al., 2013). The factor loading values of items were above 0.4 (ranging between 0.43 and 0.88), so all of the items remained in the scale. The Cronbach’s alpha and CR coefficients demonstrate acceptable internal reliability of this scale. Additionally, the AVE coefficients of the two factors of the IU-12 scale demonstrated suitable convergent validity for the measure.

A Pearson correlation analysis was utilized to assess concurrent validity with the DAS-21 and PSWQ (Meyer et al., 1990). Results demonstrated that greater levels of inhibitory anxiety and prospective anxiety were positively associated with worry, stress, anxiety, and depression. These findings are consistent with our hypothesis and prior research (Carleton et al., 2007; Gentes and Ruscio, 2011; Nekić and Mamić, 2019; Bakioğlu et al., 2020; Wilson et al., 2020). Findings supported the relationship between IU and negative emotional states, as well as the transdiagnostic nature of the IU among university students. Uncertainty about a stimulus or situation instigates potential interpretations and responses, including the catastrophic appraisal and generalized negative prediction about future events (Liao and Wei, 2011). For example, if a person with panic disorder is certain that a physical symptom is not threatening, anxiety is less likely. Additionally, repetitive and intrusive negative thinking is a common feature of anxiety and depression. In anxiety disorders, repetitive negative thinking in the form of worry is used as a means of controlling feelings of uncertainty and anxiety about future events (Freeston et al., 1994; Liao and Wei, 2011). Similarly, a high level of rumination in people with depression intensifies negative responses to uncertain situations which in turn strengthens the belief in the occurrence of distressing events (Freeston et al., 1994; Liao and Wei, 2011).

The IU-12 is a valid and reliable measure to assess IU in university students. The short form IU-12 in comparison to the original IU-27 facilitates the evaluation of IU in various clinical and non-clinical populations. These findings have several implications. Given the satisfactory psychometric properties of the Persian version of the IU-12 scale, it can be used in various research and clinical settings to assess psychological symptoms in undergraduate students. The development of a valid and reliable scale to measure IU may contribute to promoting IU-focused interventions. Additionally, consistency in measuring IU will assist in fostering transdiagnostic models that can lead to efficient theoretical models and more treatments that are effective.

## Limitations and Future Research

Limitations of the present study underscore future implications for further research. First, this study was conducted on a sample of non-clinical university students, which reduces the generalizability of findings to clinical samples, as well as other age groups. Future research should evaluate the strength of this scale in measuring IU among different age groups and clinical samples. Future studies should also compare clinical and non-clinical samples in a single study to determine if clinical samples demonstrate the same two-factor structure of the IU-12. Second, this study used measures of anxiety, depression, stress, and worry. In order to clarify the transdiagnostic nature of IU, future research should use other measures to illustrate the relationship between IU and other psychopathologies, such as obsessive-compulsive disorder (OCD) symptoms.

## Conclusion

This study provided a precise psychometric assessment of the Persian version of the IU-12 among a non-clinical sample of Iranian university students. A confirmatory factor analysis supported that the structure of the translated IU-12 scale with two factors and analysis of its measurement properties found evidence of good psychometric properties. This measure can be served as an efficacious tool in assessing IU among Iranian university students.

## Data Availability Statement

The original contributions presented in the study are included in the article/supplementary material, further inquiries can be directed to the corresponding authors.

## Ethics Statement

The studies involving human participants were reviewed and approved by the Ethics Committee of the Alzahra University (IR/10/27/1398). The patients/participants provided their written informed consent to participate in this study.

## Author Contributions

AAbd, ZA, MT, DM, and WS collected and analyzed the data as well as prepared the manuscript. AAbb, MS, and AH analyzed the data, prepared the tables and figures, and wrote some parts of analyses sections. MS, KA, and IP reviewed and edited the manuscript and interpreted the result of data analyses. All authors contributed to the article and approved the submitted version.

## Conflict of Interest

The authors declare that the research was conducted in the absence of any commercial or financial relationships that could be construed as a potential conflict of interest.

## Publisher’s Note

All claims expressed in this article are solely those of the authors and do not necessarily represent those of their affiliated organizations, or those of the publisher, the editors and the reviewers. Any product that may be evaluated in this article, or claim that may be made by its manufacturer, is not guaranteed or endorsed by the publisher.

## References

[B1] AbdollahiA.HosseinianS.PanahipourH.AllenK. A. (2019). Cognitive behavioural therapy as an effective treatment for social anxiety, perfectionism, and rumination. *Curr. Psychol.* 40 4698–4707.

[B2] American Psychiatric Association (2013). *DSM V. Diagnostic and Statistical Manual of Mental Disorders (DSM-5)*, 5th Edn. Washington, DC: American Psychiatric Association.

[B3] AntonyM. M.CoxB. J.EnnsM. W.BielingP. J.SwinsonR. P. (1998). Psychometric properties of the 42-item and 21-item versions of the Depression Anxiety Stress Scales in clinical groups and a community sample. *Psychol. Assess.* 10 176–181.

[B4] AsghariA.SaedF.DibajniaP. (2008). Psychometric properties of the Depression Anxiety Stress Scales-21 (DASS-21) in a non-clinical Iranian sample. *Int. J. Psychol.* 2 82–102.

[B5] BakioğluF.KorkmazO.ErcanH. (2020). Fear of COVID-19 and positivity: mediating role of intolerance of uncertainty, depression, anxiety, and stress. *Int. J. Ment. Health Addict.* 19 2369–2382. 10.1007/s11469-020-00331-y 32837421PMC7255700

[B6] BentlerP. M.WuE. J. C. (2005). *EQS 6.1 for Windows.* Encino, CA: Multivariate Software INC.

[B7] BirrellJ.MearesK.WilkinsonA.FreestonM. (2011). Toward a definition of intolerance of uncertainty: a review of factor analytical studies of the Intolerance of Uncertainty Scale. *Clin. Psychol. Rev.* 31 1198–1208. 10.1016/j.cpr.2011.07.009 21871853

[B8] BlancoC.OkudaM.WrightC.HasinD. S.GrantB. F.LiuS. M. (2008). Mental health of college students and their non-college-attending peers: results from the national epidemiologic study on alcohol and related conditions. *Arch. Gen. Psychiatry* 65 1429–1437. 10.1001/archpsyc.65.12.1429 19047530PMC2734947

[B9] BoelenP. A.LenferinkL. I. M. (2018). Latent class analysis of indicators of intolerance of uncertainty. *Scand. J. Psychol.* 59 243–251. 10.1111/sjop.12440 29582434

[B10] BoswellJ. F.Thompson-HollandsJ.FarchioneT. J.BarlowD. H. (2013). Intolerance of uncertainty: a common factor in the treatment of emotional disorders. *J. Clin. Psychol.* 69 630–645. 10.1002/jclp.21965 23381685PMC3712497

[B11] BredemeierK.McColeK.LutherL.BeckA. T.GrantP. M. (2019). Reliability and validity of a brief version of the intolerance of uncertainty scale in outpatients with psychosis. *J. Psychopathol. Behav. Assess.* 41 221–234.

[B12] BrislinR. W. (1986). “The wording and translation of research instruments,” in *Field Methods in Cross-Cultural Research*, eds LonnerW. J.BerryJ. W. (Beverly Hills, CA: Sage), 137–164.

[B13] ByrneB. M. (2013). *Structural Equation Modeling With Mplus: Basic Concepts, Applications, and Programming.* London: Routledge.

[B14] CarletonR. N. (2016). Into the unknown: a review and synthesis of contemporary models involving uncertainty. *J. Anxiety Disord.* 39 30–43. 10.1016/j.janxdis.2016.02.007 26945765

[B15] CarletonR. N.FetznerM. G.HacklJ. L.McEvoyP. (2013). Intolerance of uncertainty as a contributor to fear and avoidance symptoms of panic attacks. *Cogn. Behav. Ther.* 42 328–341. 10.1080/16506073.2013.792100 23758117

[B16] CarletonR. N.NortonM. A. P. J.AsmundsonG. J. G. (2007). Fearing the unknown: a short version of the Intolerance of Uncertainty Scale. *J. Anxiety Disord.* 21 105–117. 10.1016/j.janxdis.2006.03.014 16647833

[B17] CookD. A.BeckmanT. J. (2006). Current concepts in validity and reliability for psychometric instruments: theory and application. *Am. J. Med.* 119 166.e7–16. 10.1016/j.amjmed.2005.10.036 16443422

[B18] DehshiriG.GolzariM.BorjaliA. (2010). Psychometrics particularity of farsi version of pennsylvania state worry questionnaire for college students. *J. Clin. Psychol.* 1 67–75.

[B19] DugasM. J. (1997). Intolerance of uncertainty and problem orientation in worry. *Cogn. Ther. Res.* 21 593–606.

[B20] DugasM. J.GagnonF.LadouceurR.FreestonM. H. (1998). Generalized anxiety disorder: a preliminary test of a conceptual model. *Behav. Res. Ther.* 36 215–226.961302710.1016/s0005-7967(97)00070-3

[B21] FergusT. A.WuK. D. (2013). The intolerance of uncertainty scale: measurement invariance, population heterogeneity, and its relation with worry among self-identifying white and black respondents. *Assessment* 20 555–564. 10.1177/1073191112460272 22984142

[B22] FreestonM. H.RhéaumeJ.LetarteH.DugasM. J.LadouceurR. (1994). Why do people worry? *Pers. Individ. Dif.* 17 791–802.

[B23] GentesE. L.RuscioA. M. (2011). A meta-analysis of the relation of intolerance of uncertainty to symptoms of generalized anxiety disorder, major depressive disorder, and obsessive-compulsive disorder. *Clin. Psychol. Rev.* 31 923–933. 10.1016/j.cpr.2011.05.001 21664339

[B24] HairJ. F.AndersonR. E.TathamR. L.BlackW. C. (1998). *Multivariate Data Analysis.* Englewood Cliffs, NJ: Prentice Hall.

[B25] HajizadehE.AsghariM. (2011). *Statistical Methods and Analyses in Health and Biosciences a Research Methodological Approach.* Tehran: Tehran Jahade Daneshgahi Publications.

[B26] HongR. Y.CheungM. W. L. (2015). The structure of cognitive vulnerabilities to depression and anxiety: evidence for a common core etiologic process based on a meta-analytic review. *Clin. Psychol. Sci.* 3 892–912.

[B27] HuntleyC. D.YoungB.Tudur SmithC.FisherP. L. (2020). Uncertainty and test anxiety: psychometric properties of the Intolerance of Uncertainty Scale – 12 (IUS-12) among university students. *Int. J. Educ. Res.* 104:101672.

[B28] JacobyR. J.AbramowitzJ. S.ReumanL.BlakeyS. M. (2015). Enhancing the ecological validity of the Beads Task as a behavioral measure of intolerance of uncertainty. *J. Anxiety Disord.* 41 43–49. 10.1016/j.janxdis.2016.02.003 26896872

[B29] JacobyR. J.FabricantL. E.LeonardR. C.RiemannB. C.AbramowitzJ. S. (2013). Just to be certain: confirming the factor structure of the Intolerance of Uncertainty Scale in patients with obsessive-compulsive disorder. *J. Anxiety Disord.* 27 535–542. 10.1016/j.janxdis.2013.07.008 23973743

[B30] KesbyA.MaguireS.BrownlowR.GrishamJ. R. (2017). Intolerance of Uncertainty in eating disorders: an update on the field. *Clin. Psychol. Rev.* 56 94–105. 10.1016/j.cpr.2017.07.002 28710918

[B31] KesslerR. C.WaltersE. E.ForthoferM. S. (1998). The social consequences of psychiatric disorders, III: probability of marital stability. *Am. J. Psychiatry* 155 1092–1096. 10.1176/ajp.155.8.1092 9699699

[B32] KhawajaN. G.YuL. N. H. (2010). A comparison of the 27-item and 12-item intolerance of uncertainty scales. *Clin. Psychol.* 14 97–106.

[B33] LawsheC. H. (1975). A quantitative approach to content validity 1. *Pers. Psychol.* 28 563–575.

[B34] LeeJ. S. (2019). Effect of resilience on intolerance of uncertainty in nursing university students. *Nurs. Forum.* 54 53–59. 10.1111/nuf.12297 30300447

[B35] LiaoK. Y. H.WeiM. (2011). Intolerance of uncertainty, depression, and anxiety: the moderating and mediating roles of rumination. *J. Clin. Psychol.* 67 1220–1239. 10.1002/jclp.20846 22052621

[B36] LovibondS. H.LovibondP. F. (1996). *Manual for the Depression Anxiety Stress Scales.* Sydney, NSW: Psychology Foundation of Australia.

[B37] MeyerT. J.MillerM. L.MetzgerR. L.BorkovecT. D. (1990). Development and validation of the penn state worry questionnaire. *Behav. Res. Ther.* 28 487–495.207608610.1016/0005-7967(90)90135-6

[B38] NekićM.MamićS. (2019). Intolerance of uncertainty and mindfulness as determinants of anxiety and depression in female students. *Behav. Sci. (Basel)* 9:135. 10.3390/bs9120135 31816849PMC6960897

[B39] OglesbyM. E.BoffaJ. W.ShortN. A.RainesA. M.SchmidtN. B. (2015). Intolerance of uncertainty as a predictor of post-traumatic stress symptoms following a traumatic event. *J. Anxiety Disord.* 41 82–87. 10.1016/j.janxdis.2016.01.005 26803928

[B40] OsmanağaoğluN.CreswellC.SnuggsS.StuijfzandS.DoddH. F. (2021). Evaluating the psychometric properties of the intolerance of uncertainty scale for children in a preadolescent sample. *J. Anxiety Disord.* 77:102343. 10.1016/j.janxdis.2020.102343 33310446

[B41] RosserB. A. (2019). Intolerance of uncertainty as a transdiagnostic mechanism of psychological difficulties: a systematic review of evidence pertaining to causality and temporal precedence. *Cogn. Ther. Res.* 43 438–463.

[B42] SweeM. B.OlinoT. M.HeimbergR. G. (2019). Worry and anxiety account for unique variance in the relationship between intolerance of uncertainty and depression. *Cogn. Behav. Ther.* 48 253–264. 10.1080/16506073.2018.1533579 30354911

[B43] TabachnickB. G.FidellL. S. (2012). *Using Multivariate Statistics: International Edition.* New York, NY: Harper & Row.

[B44] TabriN.ElliottC. M. (2012). Principles and practice of structural equation modeling. *Can. Grad. J. Sociol. Criminol.* 1:59.

[B45] WhitingS. E.JenkinsW. S.MayA. C.RudyB. M.DavisT. E.ReutherE. T. (2014). The role of intolerance of uncertainty in social anxiety subtypes. *J. Clin. Psychol.* 70 260–272. 10.1002/jclp.22024 23843207

[B46] WilsonE. J.StapinskiL.DueberD. M.RapeeR. M.BurtonA. L.AbbottM. J. (2020). Psychometric properties of the Intolerance of Uncertainty Scale-12 in generalized anxiety disorder: assessment of factor structure, measurement properties and clinical utility. *J. Anxiety Disord.* 76:102309. 10.1016/j.janxdis.2020.102309 33002756

[B47] WrightK. D.LebellM. A. N. A.CarletonR. N. (2016). Intolerance of uncertainty, anxiety sensitivity, health anxiety, and anxiety disorder symptoms in youth. *J. Anxiety Disord.* 41 35–42. 10.1016/j.janxdis.2016.04.011 27302203

